# Quantitative Detection of Gastrointestinal Tumor Markers Using a Machine Learning Algorithm and Multicolor Quantum Dot Biosensor

**DOI:** 10.1155/2022/9022821

**Published:** 2022-09-01

**Authors:** Gaowa Saren, Linlin Zhu, Yue Han

**Affiliations:** ^1^The Department of Medical Nursing, Hulunbuir Vocational Technical College, Hulunbuir 021000, China; ^2^Department of Pathology, Hulunbeir People's Hospital, Hulunbuir 021008, China; ^3^Department of Endoscopy, Hulun Buir Weikang Digestive Hospital, Hulunbuir 021000, China

## Abstract

This work was to explore the application value of gastrointestinal tumor markers based on gene feature selection model of principal component analysis (PCA) algorithm and multicolor quantum dots (QDs) immunobiosensor in the detection of gastrointestinal tumors. Based on the PCA method, the neighborhood rough set algorithm was introduced to improve it, and the tumor gene feature selection model (OPCA) was established to analyze its classification accuracy and accuracy. Four kinds of coupled biosensors were fabricated based on QDs, namely, 525 nm Cd Se/Zn S QDs-carbohydrate antigen 125 (QDs525-CA125 McAb), 605 nm Cd Se/Zn S QDs-cancer antigen 19-9 (QDs605-CA19-9 McAb), 645 nm Cd Se/Zn S QDs-anticancer embryonic antigen (QDs 645-CEA McAb), and 565 nm Cd Se/Zn S QDs-anti-alpha-fetoprotein (QDs565-AFP McAb). The quantum dot-antibody conjugates were identified and quantified by fluorescence spectroscopy and ultraviolet absorption spectroscopy. The results showed that the classification precision of OPCA model in colon tumor and gastric cancer datasets was 99.52% and 99.03%, respectively, and the classification accuracy was 94.86% and 94.2%, respectively, which were significantly higher than those of other algorithms. The fluorescence values of AFP McAb, CEA McAb, CA19-9 McAb, and CA125 McAb reached the maximum when the conjugation concentrations were 25 *µ*g/mL, 20 *µ*g/mL, 30 *µ*g/mL, and 30 *µ*g/m, respectively. The highest recovery rate of AFP was 98.51%, and its fluorescence intensity was 35.78 ± 2.99, which was significantly higher than that of other antigens (*P* < 0.001). In summary, the OPCA model based on PCA algorithm can obtain fewer feature gene sets and improve the accuracy of sample classification. Intelligent immunobiosensors based on machine learning algorithms and QDs have potential application value in gastrointestinal gene feature selection and tumor marker detection, which provides a new idea for clinical diagnosis of gastrointestinal tumors.

## 1. Introduction

Tumors are caused by abnormal tissue growth caused by genetic mutations and other factors, and malignant tumors are often referred to as cancers. They invade and destroy surrounding tissue, can lead to metastasis and abnormal growth, and, if left untreated, can pose a huge threat to human health. The accurate and reliable classification of tumors is the key to the successful diagnosis and treatment of cancer [1]. In recent years, with the successful application of feature selection in bioinformatics, especially in the face of many high-dimensional data classification tasks, it has shown ideal performance [2, 3]. However, due to the complexity and variability of gene expression profile datasets and “dimension disaster” and other problems, tumor characteristic gene selection algorithms generally have shortcomings such as high computational complexity and low classification accuracy [4]. Principal component analysis (PCA) is an optimal orthogonal transformation based on the statistical properties of the target. It is the best transformation because it has important good properties. The new components generated after the transformation are orthogonal or irrelevant, and some new components represent the minimum mean square error of the original vector. After transformation, the vector becomes more determinate, and the energy is more concentrated, which makes it very important in feature extraction and data compression. Some studies have pointed out that PCA simply reduces the spatial dimension in the process of feature gene selection without considering the correlation between features and categories, which is a blind feature selection method [5] and therefore needs to be further optimized.

Gastrointestinal tumors mainly include esophageal cancer, gastric cancer, and colorectal cancer and are one of the common malignant tumors in humans. The global incidence of gastrointestinal tumors accounts for approximately 20% of all tumors [6], of which 35% of patients with malignant tumors die because of intestinal tumors, and the prognosis is poor [7]. In China, the proportion of patients who died of gastrointestinal tumors ranks among the top five in malignant tumors [8]. At present, the diagnosis of gastrointestinal tumors mainly uses imaging methods such as endoscopy, air-barium double contrast, computed tomography (CT), and magnetic resonance imaging (MRI). The pathological diagnosis result is used as the gold standard, but there are certain limitations in the diagnosis of early latent cancer under imaging and pathology [9]. With the continuous research of molecular biology and tumor molecular mechanisms in recent years, tumor marker detection has been used as an effective means of gastrointestinal cancer diagnosis because of its low cost, noninvasiveness, and simple operation [10]. Tumor marker detection can effectively identify benign and malignant diseases and tumor staging and can also detect tumor recurrence and metastasis [11].

Carcinoembryonic antigen (CEA) is a protein complex rich in polysaccharides. Current research results have found that, under normal circumstances, CEA in the body can be metabolized through the gastrointestinal tract. Once a gastrointestinal tumor occurs, CEA metabolism in the body will be abnormal, which will lead to a significant increase in the CEA content in the body [12]. At present, CEA has been used as a tumor marker for a variety of cancers, such as colorectal cancer, gastric cancer, lung cancer, and breast cancer, and it plays an important role in early tumor screening. Carbohydrate antigen 125 (CA125) is a group of high-molecular-weight glycoproteins mainly found in the epithelial cells of the digestive tract, the endothelium of the pleural oviduct, and the endocervical lining [13]. At present, CA125 is mainly used in the diagnosis and screening of ovarian cancer. In recent years, a large number of research results have pointed out that the levels of CA125 in cancer patients, such as those with gastric cancer, colorectal cancer, and breast cancer, have increased to varying degrees [14]. Cancer antigen 19-9 (CA19-9) is a monosialic acid ganglioside. A large number of studies have shown that the levels of CA19-9 in patients with adenocarcinoma, gastric cancer, and colorectal cancer are significantly increased [15]. At present, CA19-9 is mainly used clinically in the auxiliary diagnosis and early screening of pancreatic cancer. Alpha-fetoprotein (AFP) is a glycoprotein whose content is extremely low in normal bodies, but its content is significantly higher in cancerous cells. It is currently mainly used in the auxiliary diagnosis of liver cancer. Studies have pointed out that the levels of AFP in the serum of cancer patients, such as gastric cancer, lung cancer, and colorectal cancer patients, are also significantly increased [16]. Positive rates of tumor markers CEA, CA125, CA19-9, and AFP in gastrointestinal tumors have been reported. Studies have pointed out that the positive rate of CEA in gastrointestinal cancer serum is approximately 40% [17], the detection rate of CA125 is approximately 15% [18], the positive rate of CA19-9 is approximately 40% [19], and the positive rate of AFP is approximately 10% [20]. The detection rates of different tumor markers are different, and the sensitivity and specificity of a single tumor marker are not high. Therefore, the combined determination of multiple markers should be used to increase the detection rate of tumors.

At present, the clinical detection methods of tumor markers mainly include ELISA, chemiluminescence immunoassays, biochip methods, and microarray methods [21]. However, these detection methods are costly, time-consuming, and labor-intensive. Lateral flow immunoassay (LFIA) is a biosensor made from materials such as cellulose or nitrocellulose. Because of its good stability, high detection sensitivity, and fast detection speed, it is widely used in many fields, such as food safety, water quality detection, and medical diagnosis [22, 23]. Quantum dots (Ds) are semiconductor nanoparticles with a particle size between 1 and 10 nm [24]. QDs have good biocompatibility and luminescence properties and are widely used in the detection of microorganisms, proteins, and nucleic acids [25]. Researchers have used QDs in immunochromatographic techniques and applied them in drug, environmental, food, and medical testing, and they found that the sensitivity of QDs to be tested is significantly improved [26]. Multiple QDs can be excited at the same time, and the emission spectra do not easily overlap [27], which lays a theoretical foundation for the combined determination of multiple markers.

In summary, PCA algorithm has significant advantages in the process of data feature extraction, but it still has limitations in gene feature extraction, which needs to be further optimized. Therefore, based on PCA calculation, the gene feature selection model was established by optimizing it, and the classification accuracy and accuracy of OPCA model based on PCA algorithm in gene feature selection were discussed, so as to provide reference for gene feature selection method selection. In addition, the combined detection of multiple markers is of great significance for tumor monitoring, and QDs have the advantage of being harnessed in immunochromatography. In this study, based on the needs of tumor detection and the advantages of QDs, a multicolor QD-labeled biofilm sensor was developed to realize the quantitative detection of multiple tumor markers and was applied to the detection of GITMs to explore the application value of QD-based multicolor biosensing films in the detection of GITMs and provide a new diagnostic method for the monitoring of gastrointestinal tumors.

## 2. Experimental Details

### 2.1. Establishment of a Tumor Gene Feature Selection Model Based on Principal Component Analysis (PCA)

*A*_1_, *A*_2_,…, *A*_p_ are set as *p*-dimensional random variables, and the covariance matrix is expressed as follows:

(1) $$\begin{array}{c} \sum ={\left(\sigma_{ij}\right)}_{pxp}=E\left[\left(A-E\left(X\right)\right){\left(A-E\left(X\right)\right)}^{T}\right]\text{.} \end{array}$$

A new variable *B* can be obtained by orthogonal transformation of variable *A*, and its expression is as follows:

(2) $$\begin{array}{c} Y_{p}=l_{p}^{T}A=l_{p1}A_{1}+l_{p2}A_{2}+\cdots +l_{pp}A_{p}\text{.} \end{array}$$

The principal component analysis covariance matrix is expressed as follows:

(3) $$\begin{array}{c} Cov\left(Y_{i},Y_{j}\right)=Cov\left(l_{i}^{T}A,l_{j}^{T}A\right)=l_{i}^{T}A_{j}^{l},j=1,2,\cdots ,p\text{,} \end{array}$$

where *l*_*i*_ represents *P* constant vectors, *i*=1,2, ⋯, *p*.

The PCA feature selection method has the disadvantage of weak gene discrimination ability in the process of feature gene selection, and its gene microarray contains many redundancies. To overcome the above shortcomings, a neighborhood rough set algorithm was introduced to optimize it, and a tumor gene feature selection model was established, which was named OPCA.

A neighborhood rough set is an iterative process in neighborhood calculation with high computational time complexity [28]. It is assumed that a gene dataset contains *Z* samples and *m* genes, and the reduction time consumption is *P*. To reduce the iterative operation, the OPCA model used principal component analysis dimensionality reduction to construct the low-dimensional feature space and then used a multineighborhood rough algorithm to screen out the better feature gene set. For a given *n*-dimensional feature space *Q*, its output covariance matrix *H* is expressed as shown in (3), and *M* represents the sample size of the input space.

(4) $$\begin{array}{c} H=\frac{1}{M}∙\overset{M}{\underset{k=1}{\sum }}x_{k}x_{k}^{T}\text{.} \end{array}$$

If *D* is the *N*-order matrix and *β* is a real number, then there is the following equation:

(5) $$\begin{array}{c} DX=\beta X\text{,} \end{array}$$

where *β* is called the eigenvalue of *D* and *X* is the eigenvector of *D*.

For a given gene dataset *G*, the radius parameter and the lower limit parameter of its attribute domain were calculated. The PCA algorithm was used to calculate the contribution rate of the gene dataset, and the gene dataset with a contribution rate greater than 1% was selected to initialize the reduced dataset and calculate the attribute domain value. The feature set was used to represent the gene attribute column in the gene dataset whose contribution rate was more than 1%. Then, the positive domain of the attribute and its importance degree were calculated, the positive domain set of the attribute was obtained, and the importance degree was judged to be greater than the lower limit parameter. According to the judgment result, the better characteristic gene set was finally output. The characteristic gene selection process of OPCA based on PCA is shown in Figure 1.

### 2.2. Validation of the Tumor Gene Feature Selection Model Based on PCA

Colon tumor (https://featureselection.asu.edu/datasets.php) and gastric cancer microarray dataset GSE54129 were selected to verify the OPCA gene feature selection model. There were 2,000 colon tumor dataset features. The positive and negative sample sizes were 22 and 40, respectively, and the gastric cancer microarray dataset GSE54129 contained 3894 features and 21 normal and 111 abnormal sample sizes, respectively. The experimental environment was CPU: AMD Athlon^TM^ II X4 645 processor; memory: 4 G; system: Windows 7; experimental software: MATLAB-R2010A and Weka-3.9.0. The OPCA model neighborhood parameters ranged from 0 to 2, and the importance lower limit was 0.01. The number of characteristic genes in both the colon tumor and gastric cancer datasets was 6, and the thresholds were 0.77 and 0.19, respectively. Under the same conditions, the number of characteristic genes in the OPCA gene feature selection algorithm established in this study was compared with the improved genetic algorithm (IGA) [29], PCA [30], and neighborhood rough set (NRS) [2]. The classification precision and classification accuracy were compared and analyzed.

### 2.3. Selection of Multicolor QDs

After chemical modification, water-soluble QDs can be covalently combined with antibodies (Ab) to form stable QD-Ab conjugates. One microliter of 525 nm, 545 nm, 565 nm, 585 nm, 605 nm, 625 nm, and 645 nm Cd Se/ZnS QDs (Ocean Nanotech, USA) was dropped onto a nitrocellulose (NC) membrane. After drying, the emission spectrum was measured at 365 nm using a spectrophotometer (Shimadzu, Japan).

### 2.4. Preparation of QD-Ab Antibody Conjugate

After 35 *μ*L of 525 nm, 565 nm, 605 nm, and 645 nm Cd Se/ZnS QDs with a concentration of 8 mol/L was added to different centrifuge tubes, certain amounts of 1-(3-dimethylaminopropyl)-3-ethylcarbodiimide hydrochloride 1-(3-(ethyliminomethylideneamino)-N, N-dimethylpropan-1-amine, hydrochloride, EDC) (American Sigma-Aldrich company) and N-hydroxysulfosuccinyl Imine (N-Hydroxysulfosuccinimide, NHS) were added to mix well. Phosphate buffer with a concentration of 0.01 mol/L was added to make the final concentrations of EDC and NHS in solutions of 0.4 mg/mL and 0.2 mg/mL, respectively, and shaken for 30 min at room temperature for activation. AFP McAb was added to the activated 565 nm Cd Se/ZnS QDs, CEA McAb was added to the activated 645 nm Cd Se/ZnS QDs, and the reaction was carried out at room temperature for 2 hours. After adding 500 *μ*L of 0.5% bull serum albumin (BSA) to react at room temperature for 1 hour, the mixture was centrifuged at 12,000 rpm/min for 30 minutes to collect the precipitate, which was washed with 0.01 M phosphate buffer 3 times. The pellet was resuspended in 0.01 M phosphate buffer containing 1% BSA, 0.01% NaN_3_, and 0.02% Tween-20 to obtain the QD-Ab antibody conjugate. The specific preparation process of the QD-Ab antibody conjugate is shown in Figure 2.

### 2.5. Exploration and Identification of Optimal Preparation Conditions for QD-Ab Antibody Conjugates

After activation, 10 *μ*L each of 565 nm and 645 nm Cd Se/ZnS QDs was added to a certain amount of phosphate buffer to adjust the pH to 5.0, 5.5, 6.0, 6.5, 7.0, 7.4, 8.0, 8.5, and 9.0. Then, 20 *μ*L of AFP McAb and CEA McAb at a concentration of 2 mg/mL was added under different pH systems to react for 2 h at room temperature. The fluorescence intensity of the QD-Ab antibody conjugate prepared under different pH conditions was measured by a fluorescence spectrophotometer.

After activation, 10 *μ*L of 565 nm and 645 nm Cd Se/ZnS QDs was taken and added to 0, 5, 10, 15, 20, 25, 30, and 35 g of AFP McAb and CEA McAb to adjust the pH of the reaction system to the optimal conditions and then react for 2 hours at room temperature. A fluorescence spectrophotometer was adopted to detect the fluorescence spectrum of each system.

After activation, 565 nm and 645 nm Cd Se/ZnS QDs were mixed with the optimal amounts of AFP McAb and CEA McAb, respectively. At the optimal pH, the solution was allowed to react at room temperature for 30 min, 60 min, 90 min, 120 min, 150 min, and 180 min. The reaction products were collected in a fluorescence spectrophotometer to detect the fluorescence intensity of the QD-Ab antibody conjugate under different reaction times.

Fluorescence spectroscopy and UV absorption spectroscopy were used to analyze the changes in light absorption before and after the coupling of Cd Se/ZnS QDs to identify whether the QD-Ab antibody conjugate was successfully prepared.

### 2.6. Preparation of QD Biosensors

The glass fiber membrane was used as the binding pad, cut into a size of 0.4 cm × 0.7 cm, and immersed in 0.01 M phosphate buffer containing 2% BSA, 1% sucrose, and 0.1% Tween-20 (pH 7.4). After it was dried at 37°C, 10 *μ*L QDs-Ab-AFP McAb coupling objects, QDs-Ab-CEA McAb coupling objects, QDs-Ab-CA125 McAb coupling objects, and QDs-Ab- CA19-9 McAb coupling objects were added dropwise and dried at 37°C in vacuum. The NC membrane was cut into a size of 0.4 cm × 2.4 cm, and the AFP McAb was diluted with 0.01 M phosphate buffer (pH 7.4) containing 1% sucrose to a final concentration of 1 mg/mL. The 2 *μ*L/cm was determined as the *T* band, and 0.5 mg/mL goat anti-mouse IgG was used as band C and dried at 4°C for use. The sample pad, bonding pad, NC membrane, and absorbent board were laminated in sequence and pasted onto a polyvinyl chloride (PVC) base plate. After drying at 4°C, four different quantum dot biosensors were obtained.

### 2.7. Quantitative Detection and Verification of the QD Biosensor

AFP and CEA were diluted with 0.01 M phosphate buffered saline (PBS) (pH = 7.4) to 0.25, 0.5, 1, 5, 10, 40, 60, 80, 100, and 120 ng/mL, respectively. The prepared QD biosensor was used to detect the fluorescence values of AFP and CEA and plotted as a curve. At the same time, the fluorescence of the QD biosensor at different concentrations was observed under a microscope in the dark.

AFP was diluted with 0.01 M PBS (pH = 7.4) to final concentrations of 70 ng/mL, 30 ng/mL, and 3 ng/mL. After 80 *μ*L of diluted AFP, the prepared QD biosensor was adopted to detect the fluorescence value, and the recovery rate of sample detection was calculated according to the standard curve.

Based on the methods introduced by Shariatifar et al. [31], cross-reaction experiments were performed with BSA, CA125, CA-19-9, CEA, and AFP to evaluate whether the test results between AFP and BSA, CA125, CA-19-9, and CEA could affect each other.

### 2.8. QDs Biosensor to Detect CEA, CA125, CA19-9, and AFP

For simultaneous detection of multiple tumor markers, QDs-Ab-CEA McAb, QDs-Ab-CA125 McAb, QDs-Ab-CA19-9 McAb, and QDs-Ab-AFP McAb should be prepared according to the abovementioned QDs-Ab antibody conjugates. Then, the corresponding antibody was added during the coating process of the detection tape and the quality control tape. For other operation steps, refer to the above steps.

### 2.9. Statistical Methods

The test data were processed using SPSS 19.0 statistical software, and the data were analyzed by one-way analysis of variance. The measurement data were expressed as the mean ± standard deviation ($\bar{x}\pm s$), and the count data were expressed as a percentage (%), using the *χ*^2^ test. *P* < 0.05 indicated that the difference was statistically significant.

## 3. Experimental Results and Analysis

### 3.1. Comparison of Tumor Gene Feature Selection Results with Different Gene Selection Algorithms

Under the same conditions, the number of feature genes, classification precision, and classification accuracy of the OPCA gene feature selection algorithm were compared with those of the IGA algorithm, PCA algorithm, and neighborhood rough set (NRS) algorithm. In Figure 3, the number of selected characteristic genes by the OPCA gene feature selection algorithm in both the colon tumor and gastric carcinoma datasets was 6, which was significantly lower than that of the other algorithms. The classification precision of OPCA in the colon tumor and gastric carcinoma datasets was 99.52% and 99.03%, and the classification accuracy was 94.86% and 94.2%, respectively. The OPCA gene feature selection algorithm selected the fewest feature genes, and its classification precision and accuracy were higher than those of the current algorithm. Therefore, the dataset of the original gene expression profile contained much redundant information. In the process of feature gene selection, the OPCA gene feature selection algorithm effectively removed redundant noise, improved the classification ability of the feature gene subset, and extracted fewer feature gene subsets. The reason was that PCA reduced the dimension of the feature space and the complexity of the neighborhood calculation. Meanwhile, the multineighborhood rough set algorithm calculated the neighborhood values of each gene through Euclidean distance, constructed neighborhood sets to calculate the approximation, and extracted the subset of feature genes based on heuristic search. The performance of gene feature extraction was improved by combining the two algorithms. The results showed that the OPCA gene feature selection algorithm was feasible and effective in the process of tumor gene feature extraction.

### 3.2. The Fluorescence Spectrum Detection Results of QDs

Water-soluble QDs have univariate excitation, and multiple emission characteristics are the basis for the analysis of multiple markers [32]. The selection principle of multicolor QDs is that the emission spectra of multiple QDs cannot overlap [33]. Spectral analysis of QDs in the range of 525∼645 nm (Figure 4) showed that there was obvious spectral overlap between QDs in the adjacent wavelength range. Therefore, wavelengths with a wavelength interval of 40 nm were selected for the experiment in this study; that is, 525 nm, 565 nm, 605 nm, and 645 nm QDs were selected as fluorescent materials for subsequent experiments. After excitation by 365 nm excitation light, nonoverlapping 525 nm, 565 nm, 605 nm, and 645 nm QDs were obtained, indicating that four tumor markers can be quantitatively detected simultaneously, which improved detection efficiency and reduced detection costs.

### 3.3. Coupling Conditions Analysis of QDs and Antibody

When QDs are adopted to label antibodies, the optimal conditions of the reaction system must be analyzed to ensure the effective activity of the antibodies [34]. The fluorescence intensity of QDs and antibody coupling were analyzed under different pH conditions (Figure 5). As the pH value increased, the fluorescence intensity of QDs coupled with antibodies first increased and then decreased, and the optimal pH values for coupling of different QDs with antibodies had certain differences. The optimal coupling pH of AFP McAb was 7.5, the optimal coupling pH values of CEA McAb and CA19-9 McAb were both 7.0, and the optimal coupling pH of CA125 McAb was 6.5.

The influence of different antibody concentrations on the fluorescence intensity of the conjugate was analyzed, and the results are illustrated in Figure 6. As the antibody concentration in the reaction system increased, the fluorescence intensity of the conjugate first increased and then stabilized. The fluorescence values of AFP McAb, CEA McAb, CA19-9 McAb, and CA125 McAb reached maximum values when the coupling concentrations were 25 *μ*g/mL, 20 *μ*g/mL, 30 *μ*g/mL, and 30 *μ*g/mL, respectively. Even if the antibody concentration is increased beyond the maximum value, the fluorescence value of the conjugate will no longer increase. The amount of antibody added has a significant impact on the performance of the conjugate and the entire biosensor [35]. If the amount of antibody in the reaction system is insufficient, it will cause a large number of unreacted sites in the conjugate, and nonspecific binding is likely to occur during the sample detection process, which will eventually lead to a false positive test result. If the amount of antibody in the reaction system is too high, the remaining antibodies that are not bound by the conjugate will reduce the sensitivity of sample detection when testing the sample [36].

The fluorescence intensity of the coupling substance was detected under different reaction times, as shown in Figure 7. Different antibodies reacted with the coupling substance, and the fluorescence intensity of the antibody coupling substance first increased and then stabilized as the reaction time increased. When the reaction time of AFP McAb and CEA McAb was 90 min, the fluorescence intensity reached the maximum, and when the reaction time of CA19-9 McAb and CA125 McAb was 120 min, the fluorescence intensity reached the maximum. The maximum fluorescence intensity indicates that the reaction has reached saturation at this time. The reaction time has a significant effect on the reaction of the antibody conjugate. If the reaction time is too short, the reaction between QDs and the antibody conjugate will be insufficient, resulting in false positive results [37]; if the reaction time is too long, the coupling efficiency will decrease.

### 3.4. Identification of QD-Antibody Conjugates

The successful combination of QDs and antibody conjugates plays an important role in the performance of QD biosensing membranes [38]. The fluorescence spectra of different antibody conjugates were analyzed before and after coupling with QDs, and the results are given in Figure 8. The fluorescence intensities of QDs525-CA125, QDs605-CA19-9, QDs645-CEA, and QDs565-AFP after binding antibodies were more enhanced than those of unconjugated QDs. It may be that the surface defect of QDs is modified after the antibody conjugate is combined with QDs, which increases the prefluorescence intensity of the QD conjugate. Moreover, there is no fluorescence peak shift after the QDs at different wavelengths are combined with the antibody conjugate [39], indicating that the QDs only bind to the antibody conjugate during the coupling process, and there is no polymerization reaction between the QDs.

Figure 9 shows the UV absorption spectra of different antibody conjugates before and after coupling with QDs. The UV absorption values of QDs525-CA125, QDs605-CA19-9, QDs645-CEA, and QDs565-AFP after binding to the antibody were all higher than those of unconjugated QDs, and the maximum absorption wavelength did not shift, indicating that the antibody conjugate and QDs were combined successfully.

### 3.5. Analysis of AFP Quantitative Detection Results

Under the optimal reaction conditions, the method established in this study was used to detect different concentrations of AFP standards. During the detection of AFP standards, the fluorescence intensity in the fluorescence image increased with increasing AFP concentration (Figure 10). The QD biosensing membrane was placed in a fluorescence reader to detect the fluorescence value of the T-band and C-band, and the AFP standard curve for multicolor QD biosensor detection was analyzed (Figure 11). With increasing AFP concentration, the T/C value of the QD biosensing film increased. The linear fitting equation of the T/C value and AFP concentration was *y* = 0.448*x* − 6.1923 (*R*^2^ = 0.9335), showing a good linear relationship.

Biosensors used in clinical applications need to have repeatable and reliable test results [40]. The actual concentration of AFP, multicolor QD biosensor detection concentration, and recovery rate were further analyzed, as illustrated in Figure 10. The actual concentration of AFP was not much different from the concentration of AFP detected by the multicolor QD biosensor. The recovery rate of AFP was up to 98.51%. The closer the sample recovery rate is to 100% and the closer the detection concentration is to the actual concentration, the higher the reliability of the biosensor is [41], indicating that the multicolor QD biosensor has higher repeatability and reliability.

To verify the specificity of the immune method of the QD biosensor for AFP detection, the QD biosensor was adopted to detect and analyze BSA, CA125, CA-19-9, CEA, and AFP nonspecific antigens (Figure 12(b)). The fluorescence intensity of AFP was 35.78 ± 2.99, which was significantly higher than those of the other antigens (*P* < 0.001). Without labeled AFP, even if the concentration of nonspecific antigen is high, a strong fluorescence value cannot be detected. This shows that when there is no labeled antigen, nonspecific antigens will not have an immune response, indicating that this method has significant specificity for detecting AFP.

### 3.6. The Results of Quantitative Detection of GITM Using the Multicolor QD Biosensor

Cross-reactivity is the main parameter for the specific evaluation of immunoassay methods [42]. For the detection of multiple tumor markers, it is necessary to analyze whether there is a cross-reaction between multiple tumor markers and the biosensor in the same space [33]. In this study, the results of quantitative detection of GITMs using a multicolor QD biosensor were analyzed, and the results are shown in Figure 13. Four independent proteins CA125, CA-19-9, CEA, and AFP were added to the multicolor QD biosensor, and the multicolor QD biosensor diluent was used as a blank control. Then, the detection of the four tumor markers showed good specificity, and there was no interference between them.

The results of single index detection and simultaneous multi-indicator detection were compared and analyzed, and the results are shown in Figure 14. Under different methods, there was no significant difference in the fluorescence intensity of the four GITMs (*P* > 0.05), indicating that the specificity of the mixed detection of the four test samples was better.

The fluorescence intensity of the multicolor QD biosensor simultaneously detecting the tumor markers CA125, CA-19-9, CEA, and AFP was analyzed at different concentrations (Figure 15). With increasing concentrations of the tumor markers CA125, CA-19-9, CEA, and AFP, the fluorescence value of the multicolor QD biosensor also showed an upward trend. This is because as the concentration of tumor markers CA125, CA-19-9, CEA, and AFP increases, more immune complexes Ds525-CA125, QDs605-CA19-9, QDs645-CEA, and QDs565-AFP are formed, and the more multicolor QD biosensor *T* had a higher fluorescence value.

The detection curve was drawn with the concentration of GITMs CA125, CA-19-9, CEA, and AFP as the abscissa and the corresponding T/C value as the ordinate. The linear equation and the corresponding detection linear region are shown in Table 1. When the four tumor markers CA125, CA-19-9, CEA, and AFP were detected by the multiquantum dot biosensor multi-index synchronous detection method, the corresponding tumor marker concentration ranges were 2.0–51.5 ng/mL, 4.5–40.0 ng/mL, 2.0–29.5 ng/mL, and 8.5–36.5 ng/mL, respectively. The confidence detection range was wide and could meet the clinical application. When the concentration was too low (<0.9 ng/mL), the detection sensitivity could also decrease [43].

## 4. Conclusion

Based on the PCA method, the neighborhood rough set algorithm was introduced to improve it, and the tumor gene feature selection model (OPCA) was established. Furthermore, an immunobiosensor based on multicolor QDs was prepared and applied to the quantitative detection of potential gastrointestinal tumor markers. The results showed that the OPCA model can obtain fewer feature gene sets and improve the accuracy of sample classification. Intelligent immunobiosensors based on OPCA model and multicolor QDs had high specificity in the detection of gastrointestinal tumor markers. However, there were still some shortcomings in this study. In this study, only standard samples were tested, not clinical samples. In the future work, clinical samples of patients with gastrointestinal cancer will be further collected, and the intelligent immunobiosensor prepared in this study will be used to detect them, so as to verify the clinical application value of the intelligent immunobiosensor based on multicolor QDs. In conclusion, the intelligent immunobiosensor based on machine learning algorithm and QDs has potential application value in gastrointestinal gene feature selection and tumor marker detection, which provides a new idea for clinical diagnosis of gastrointestinal tumors.

## Figures and Tables

**Figure 1:** Flow chart of characteristic gene selection based on OPCA.

**Figure 2:** Flow chart of the preparation of the QD-Ab antibody conjugate.

**Figure 3:** Comparison of tumor gene feature selection results with different gene selection algorithms. (a) Comparison of the number of tumor gene characteristics with different gene selection algorithms; (b) comparison of precision of tumor gene feature selection by different gene selection algorithms; (c) comparison of accuracy of tumor gene feature selection by different gene selection algorithms.

**Figure 4:** Emission spectra of QDs at different wavelengths.

**Figure 5:** Fluorescence intensity change curve of the conjugate under different pH values.

**Figure 6:** The effect of antibody concentration on the fluorescence intensity of the coupling reaction system.

**Figure 7:** The effect of reaction time on the fluorescence intensity of the coupling reaction system.

**Figure 8:** Fluorescence spectrum of QDs. (a) Fluorescence spectra of QDs525 and antibody conjugate before and after reaction; (b) fluorescence spectra of QDs565 and antibody conjugate before and after reaction; (c) fluorescence spectra of QDs605-CA19-9 and antibody conjugate before and after reaction; (d) fluorescence spectra before and after the reaction between QDs645-CEA and antibody conjugate.

**Figure 9:** UV absorption spectrum of QDs. (a) UV absorption spectrum before and after the reaction of QDs525 with antibody conjugate; (b) UV absorption spectrum before and after reaction of QDs565 with antibody conjugate; (c) UV absorption spectrum before and after reaction of QDs605-CA19-9 with antibody conjugate; (d) UV absorption spectra before and after the reaction between QDs645-CEA and the antibody conjugate.

**Figure 10:** AFP fluorescence image detected by QDs sensor.

**Figure 11:** AFP standard curve based on the multicolor QD biosensor.

**Figure 12:** Analysis of AFP standard test results. (a) Recovery test result of AFP standard product; (b) detection specificity of AFP.

**Figure 13:** Quantitative detection of GITM-specific analysis using a multicolor QD biosensor.

**Figure 14:** Analysis of the results of single index detection and multi-indicator simultaneous detection.

**Figure 15:** The fluorescence spectra of CA125, CA-19-9, CEA, and AFP simultaneously detected by the multicolor QD biosensor.

**Table 1:** Linear area table of simultaneous multi-indicator detection using the multiple QD biosensor.

Tumormarkers	Standard curve line	Linear workingarea (ng/mL)	*R* ^2^
CA125	*y* = 0.2248*x* − 3.7298	2.0∼51.5	0.9884
CA-19-9	*y* = 0.1658*x* + 2.4854	4.5∼40.0	0.9756
CEA	*y* = 0.1262*x* − 3.3665	2.0∼29.5	0.9637
AFP	*y* = 0.1135*x* + 6.9125	8.5∼36.5	0.9601

## Data Availability

All data are fully available without restriction.
